# Network Security Problems and Countermeasures of Hospital Information System after Going to the Cloud

**DOI:** 10.1155/2022/9725741

**Published:** 2022-07-18

**Authors:** Shuming Gao

**Affiliations:** Information Department, Pingdu People's Hospital, No. 112, Yangzhou Road, Pingdu, Shandong 266700, China

## Abstract

In the current social context, information technology, network technology, and cloud computing have been widely used in all walks of life. The analysis of the specific application results of progressive technology shows that the use of technology has changed the working state of various industries and improved the work efficiency and quality of the industry. It should be noted that although the application of some technologies will bring many positive belongings, the potential risks brought by them cannot be ignored. As far as the hospital is concerned, the information system using cloud computing technology can make better use of the hospital's information data, but after the information system is on the cloud, new problems will appear in network security, resulting in the leakage of hospital patient information or research information. Based on this, in practice, it is necessary to analyze the network security problems after the hospital information system goes to the cloud and build and implement the corresponding strategies. The author analyzes and discusses the corresponding contents through work practice and combined with previous articles, in order to provide guidance and help for peers.

## 1. Introduction

Under the environment of the continuous development of network technology and the widespread use of mobile terminals, the application of network technology is becoming more and more common. According to the current data summary, the use of the Internet has changed the working state of all walks of life, solved many problems between information transmission and the connection of things, and achieved great changes in social life. It should be noted that the widespread use of the Internet brings not only the convenience of life and work but also some security issues, such as information leakage. Therefore, in the process of network application, it is of great significance to analyze and discuss related problems and emphasize the countermeasures to solve the problems [1–3]. Through the analysis of the current development of the hospital, the hospital information system stores, transmits, and utilizes a large amount of data, especially with the rise of Internet hospitals, and many hospitals begin to use cloud computing technology. It greatly improves the patient's medical experience, but while the convenience of the hospital information system is brought by the cloud, new network security problems will also arise. Therefore, we analyze the network security problems after the hospital information system is connected to the cloud and provide countermeasures to solve the problem. The discussion has outstanding practical value.

## 2. Comparison of the Network Architecture before and after the Hospital Information System Goes to the Cloud

Comparing and analyzing the network structure of the hospital information system before and after going to the cloud have outstanding practical implication for a more specific analysis of the security network security difficulties after going to the cloud. The following is a comparative study of the information system of a tertiary hospital in China before and after the cloud.

### 2.1. Original Network Architecture

Figure 1 shows the original network architecture, and its basic operating mechanism is as follows:

1. The terminals in the hospital are divided into dissimilar VLANs, and the gateways are all on the core switch
2. Configure the NAT policy and port mapping of some terminals on the egress firewall. Only the external network segment and some servers that need to access the Internet can go to the Internet through the firewall
3. The egress firewall is also configured with an access control policy to block the traffic of known dangerous ports and restrict the server to only service ports that can pass through the firewall [4, 5]
4. Connect IPS intrusion prevention equipment in series between the egress firewall and the core switch to detect and block attacks
5. Configure ACL on the core switch to restrict the terminal in the hospital from accessing the management port of the network device and restrict the terminal from connecting to the service server through the remote desktop
6. Configure ACL on the server aggregation switch to restrict access to server file sharing ports
7. The server aggregation switch is connected to the IDS intrusion detection device to detect the interactive traffic between the server and the terminals in other areas and optimize and adjust the security policy of the equipment in each area according to the situation
8. Due to the limitations of the egress firewall NAT policy and port mapping, intranet terminals and most servers that are not within the scope of address translation and port mapping cannot interrelate with the Internet through the egress firewall

### 2.2. Network Architecture after Going to the Cloud

Figure 2 shows the cloud network architecture, and its operating mechanism is as follows:

1. The egress firewall has its own IPS function; so, the IPS device is removed
2. All office network segments in the hospital are configured with address translation. By configuring the access control policy, the original intranet terminal can only access the cloud server domain name through the DNS server equipped in the intranet, and the external network terminal can access the domain name except for the access control policy and blacklist. Other internet addresses and ports outside the restrictions
3. The intranet DNS server only configures the mapping relationship between cloud service IP addresses and domain names [6]
4. The security configuration rules of core switches and server aggregation switches are the same as before

### 2.3. Comparative Analysis of Architecture

Comparing the original structure and the cloud structure, there are the following differences:

1. After the cloud service is opened, the network architecture remains basically unchanged. The external network terminals, servers that need to access the Internet, and servers that need to be mapped to the outside still maintain the original security control policy, which is consistent with the experience before the cloud service goes online
2. Intranet terminals, DNS servers, and servers that were originally unable to access the Internet, after the cloud service goes online, set up address translation on the egress firewall, cooperate with the access control security policy, black, and white list functions, and can only access the necessary cloud server addresses and business port
3. The egress firewall has the IPS function, which is used to block external network attacks against the internal network, and the original IPS equipment is removed from the shelf
4. The security policy and blacklist configured on the egress firewall control the traffic interaction of dangerous ports between all internal terminals and external terminals
5. The egress firewall is changed from the original one to two, and the reliability of the egress device is enhanced through the hot backup function
6. The core switch and server aggregation switch keep the original port access control policy unchanged, still restrict the terminal's management of network devices, and limit the connection of remote desktop ports and file sharing ports
7. The security policy on the cloud server side is the responsibility of the relevant cloud operator, but its security information must be carefully checked

The paper arrangements are as follows: Section 2 discusses the network security problems and solutions after the hospital information system is migrated to the cloud.  Section 3 analyzes the change the concept and pay attention to network security issues.  Section 4 evaluates the building a network security system based on the actual needs of network security.  Section 5 examines the emphasis on network security management.  Section 6 concludes the article.

## 3. Network Security Problems and Solutions after the Hospital Information System Is Migrated to the Cloud

The main security problems after the hospital information system is migrated to the cloud are reflected in two aspects:

1. Information data leakage [7, 8]: the first problem after the hospital information system goes to the cloud is the leakage of information data. All hospital information is transmitted on the Internet. As far as hospital information and data are concerned, on the one hand, there is a large amount of patient information in the hospital. Once the data is leaked, it will lead to the disclosure of patient privacy, which is not good for the patient itself, and will also cause the patient to feel uncomfortable. The crisis of trust in the hospital is very unfavorable for alleviating the contradiction between doctors and patients. On the other hand, there is a large amount of disease research data in hospitals. If these data related to disease research are used properly, they will benefit society. If they are stolen by criminals or hostile elements, it is likely to cause social disasters and even endanger national security. So, the impact of a hospital research data breach is huge
2. Information data is lost or damaged [9, 10]: a large amount of information and data of a hospital has its value; so, the data of a hospital is one of the rare assets of a hospital. If the database resources are lost or the data resources are damaged and cannot be recovered due to network problems, the related work of the hospital will be greatly affected, which is not conducive to the stable and sustainable development of the hospital's scientific research work and other work. Analyze and solve such problems. Faced with the security problems that exist after the hospital information system is migrated to the cloud, security protection measures should be deployed from the following aspects

## 4. Change the Concept and Pay Attention to Network Security Issues

Based on the analysis of practice, it can be seen that in the past hospital management practice, an important reason for the frequent occurrence of network security problems is that the hospital ignores the importance of network security in the process of using information systems; so, many work arrangements exist. There are omissions in cybersecurity [11–13]. Based on this, it is necessary to change cognition and pay attention to network security. As far as the current work practice is concerned, in order to change the perception of network security, the following work needs to be done:

1. Strengthen the discussion of network security issues and explain the practical value of network security. In the utilization practice of hospital information system, an significant reason why network security is neglected is that staff does not realize the value of network security. By making the staff aware of the value of network security through discussion, they will pay more attention to network security
2. Analyze the relevant elements of network security. In the practice of hospital network security, some staff is aware of the importance of network security, but they do not systematically recognize the influencing factors of network security; so, there is a one-sided phenomenon in the process of network security work organization and implementation. Based on this, in the organization and development of network security work, strengthen research and discussion and clarify the elements related to network security, so that the organization and development of network security work will be more targeted and effective. In short, through in-depth analysis to clarify the cognition of network security, this can provide theoretical guidance for the current hospital network security work

## 5. Building a Network Security System Based on the Actual Needs of Network Security

From the point of view of the network security after the hospital information system is migrated to the cloud, in order to truly prevent network security problems, it is necessary to formulate a security structure that has a protective effect on the hospital information system based on the current state of network security. As far as the construction of safety structure is concerned, the following contents need to be emphasized:

1. Basic investigation [14]: the so-called basic investigation mainly refers to the detailed investigation of the hospital information system. In the detailed investigation of the hospital information system, it is necessary to clarify the different data partitions of the information system, such as which databases exist in the information system and what is the specific application purpose of the database, which needs to be emphasized in the investigation. Because the application value of the database is obtained based on the investigation, it can provide a reference for the determination of the security level of the database within the information system
2. Determination of the security level of the information system [15]: under the guidance of basic survey data, the internal database of the information system and the use value of the data are analyzed, and the security level is evaluated. In this way, the security level evaluation result can provide a reference for the design and construction of the network security structure of the information system
3. Construction of network security structure based on security evaluation level [16]: based on the evaluation results, it can be seen that different data security levels have different requirements. Therefore, in the construction of the security structure, the multilayer protection structure is used as the security protection structure of the core database. Important databases, general databases, etc. can build a three-layer protection structure, or it is a two-layer protective structure to protect it safely. To put it simply, based on the actual needs of network security, a targeted network security protection structure is constructed, so that the security protection effect of the hospital information system will be significantly improved

## 6. Emphasis on Network Security Management

The so-called management improvement refers to the use of management measures to avoid or stop the occurrence of network security problems. In terms of management strengthening, the main measures are as follows:

1. System improvement [17]: the implementation of specific safety management work needs to be supported by a sound system, so that the effectiveness and pertinence of the work implementation will be more prominent. As far as the current management of hospital information systems is strengthened, on the one hand, it is necessary to formulate a comprehensive responsibility system and clarify the responsibility for network security management. In this way, the implementation of management work will be more prominent. On the other hand, it is to instrument the supervision system, that is, to supervise the specific implementation of network security management work to confirm the actual effect of the work, so that network security problems can be effectively solved
2. Technological innovation [18]: the so-called technological innovation mainly refers to the use of advanced technology to reform the current network security management in the practice of network security management, so that the specific implementation of network security management will show more significant effects
3. Introduce an early warning mechanism in the process of network security management, which is, set up an alarm system in the network security structure and trigger the warning system when information leakage or other security problems occur, so that managers can timely discover network security loopholes and problem and deal with it. In this way, the adverse effects of network security issues in hospital information systems will be effectively dealt with [19, 20]

## 7. Conclusion

To sum up, the management of the hospital information system has a significant impact on the specific development of hospital work; so, it is necessary to strengthen the management of the hospital information system in practice. Based on the analysis of the current hospital practice, it can be seen that the hospital information system will face more significant network security problems after going to the cloud. Therefore, the article analyzes the performance and causes of the network security problems after the hospital information system goes to the cloud. At the same time, it discusses the countermeasures; the purpose is to guide practice.

## Figures and Tables

**Figure 1:** Original network architecture.

**Figure 2:** Cloud network architecture.

## Data Availability

The dataset used in this paper are available from the corresponding author upon request.
